# Clinical Efficacy Analysis of Fast Rehabilitation Nursing on Pain Mitigation after Lumbar Discectomy and Bone Graft Fusion and Internal Fixation

**DOI:** 10.1155/2022/3665919

**Published:** 2022-07-09

**Authors:** Lingling Fang

**Affiliations:** Department of Orthopedics First Ward, Lu'an Hospital of Anhui Medical University, Lu'an People's Hospital of Anhui Province, Lu'an, China

## Abstract

**Objective:**

To investigate clinical efficacy analysis of fast rehabilitation nursing on pain mitigation after lumbar discectomy and bone graft fusion and internal fixation.

**Methods:**

A total of 60 patients with lumbar disc herniation who underwent lumbar discectomy and bone graft fusion and internal fixation in our hospital from January 2021 to December 2021 were randomized either into routine group (*n* = 30) or rehabilitation group (*n* = 30) via the random number table method. The patients in the routine group were intervened with the routine postoperative nursing mode, and the patients in the rehabilitation group were intervened with the fast rehabilitation nursing mode on the basis of the nursing of the patients in the routine group. The rehabilitation effect, self-rating anxiety scale (SAS) and self-rating depression scale (SDS) scores, postoperative pain improvement, and nursing satisfaction were compared between the two groups.

**Results:**

The postoperative rehabilitation effect of the rehabilitation group was significantly better than that of the routine group (*P* < 0.05). The fast rehabilitation nursing resulted in a notably lower postoperative SAS and SDS scores versus the routine nursing (*P* < 0.001). The postoperative pain was significantly mitigated in the rehabilitation group when compared with the routine group (*P* < 0.001). The fast rehabilitation nursing implemented in the rehabilitation group led to a remarkably higher nursing satisfaction of the patients (*P* < 0.001).

**Conclusion:**

The fast rehabilitation nursing mode intervention for lumbar disc herniation patients undergoing lumbar discectomy and bone graft fusion and internal fixation is a promising approach to improve the postoperative rehabilitation, mitigate postoperative pain, and relieve anxiety, depression, and other negative emotions, with higher clinical nursing satisfaction.

## 1. Introduction

Lumbar intervertebral disc herniation is a common lumbar intervertebral disc rupture disease in clinical orthopaedics. It is the result of the rupture of the annulus fibrosus, which causes the nerve root of the patient to be compressed by the nucleus pulposus and then leads to the occurrence of lumbar intervertebral disc herniation [1]. With the rapid economic development in recent years, the loaded work and life pressure gives rise to the incidence of lumbar disc herniation [2]. The clinical manifestations of patients with lumbar intervertebral disc herniation are mainly waist and leg pain and even may be unable to stand in severe cases [3]. Clinically, patients with lumbar disc herniation are treated by surgery. Relevant studies have shown that lumbar discectomy and bone graft fusion and internal fixation can effectively mitigate the pain in patients with lumbar disc herniation. It also features low trauma, fast recovery, and simple operation [4], which makes the surgical method widely favored by patients and physicians. However, due to the lack of understanding of the knowledge of their own diseases in most patients, patients are prone to resistance to treatment, and it greatly compromises the effect of the operation [5].

In the context of the continuous transformation of biomedical models, perioperative care for lumbar spine diseases is not limited to the regulation and implementation of the nursing work system, but also involves how to promote the speed of postoperative recovery and improve the quality of life of patients. Simultaneously, with the continuous improvement of people's living standards and the level of medical and health knowledge, people's requirements for medical services are getting higher and higher. The fast recovery surgery nursing model is an emerging type of nursing method. On the basis of evidence-based medicine, patients are given perioperative optimization nursing intervention. Through the discussion of the nursing team, the routine perioperative nursing measures are improved, optimized to reduce the patient's stress response and maintain the balance of the patient's body indicators [6, 7]. Additionally, the fast recovery surgical nursing model can dynamically evaluate the patient's condition, timely optimize the nursing work content according to the patient's condition change and nursing needs, and promote the effective recovery of the patient's disease [8–10]. In addition, compared with routine nursing, the fast recovery surgical nursing model can integrate the advantages of multidisciplinary participation, improve the nursing intervention system, break the limitations of nursing work content, and effectively provide patients with more scientific care. It can greatly improve the patient's satisfaction with medical services and reduce the occurrence of adverse reactions of patients and provide patients with safer nursing intervention. Coombe et al. [6] pointed out that aggressive and effective nursing intervention for patients with lumbar disc herniation who underwent lumbar discectomy and bone graft fusion and internal fixation is of great significance for improving the postoperative recovery of patients. To that end, this study aimed at exploring the effect of fast rehabilitation nursing on pain relief in patients with lumbar discectomy and bone graft fusion and internal fixation.

## 2. Materials and Methods

### 2.1. Patients

A total of 60 patients with lumbar disc herniation who underwent lumbar discectomy and bone graft fusion and internal fixation in our hospital from January 2021 to December 2021 were randomized either into routine group (*n* = 30) or rehabilitation group (*n* = 30) via the random number table method. There were 27 males and 13 females in the routine group; the mean age was (52.43 ± 2.35) years; the mean disease duration was (10.53 ± 1.26) months. There were 28 males and 12 females in the rehabilitation group; the average age was (52.51 ± 2.36) years; the average disease duration was (10.48 ± 1.32) months. The two group patients presented similar baseline data. This study has been reviewed and approved by the Medical Ethics Committee of the Lu'an Hospital of Anhui Medical University (approval no. 1669-12).

### 2.2. Inclusion and Exclusion Criteria

Inclusion criteria: (1) the patients were diagnosed with lumbar disc herniation by clinical examination; (2) the cognitive and communication ability of the patients were normal; (3) all patients were informed of the study and signed an informed consent. Exclusion criteria: (1) patients with severe heart, liver, and other organic dysfunction; (2) patients with abnormal coagulation function; (3) patients with severe neurological diseases or cognitive impairment.

### 2.3. Methods

Patients in the routine group were given routine nursing intervention, including life guidance, dietary guidance, psychological counseling, and health education. The patients in the rehabilitation group were combined with the nursing intervention of fast rehabilitation on the basis of the nursing of the patients in the routine group, while integrating traditional Chinese medicine intervention. (1) Pain care: in the postoperative care of the patients, the degree of pain of the patients should be evaluated first. At the same time, it is necessary to ensure that the environment of the ward is clean and comfortable, so as to improve the feeling of comfort of the patient, which is conducive to reducing pain; moreover; it is necessary to play light music for the patient, chat with the patient, and give the patient psychological support and counseling to distract the patient's attention to achieve the purpose of pain relief [7]. (2) Straight leg raising training: after the patient's drainage tube is pulled out, the straight leg raising exercise should be performed as soon as possible with a gentle force within the patient's tolerance. The patient's surgical incision is easily stretched and causes pain, and pain care needs to be strengthened; with the gradual recovery after surgery, the pain can be gradually relieved. At this moment, the patient can gradually increase the straight leg raising force and the frequency of exercises. (3) Rehabilitation guidance: starting from day 3 after the operation, the patient should be guided and assisted in standing, walking, and other exercises, in a gradually prolonged duration manner; day 5 to 7 after the operation, according to the patient's recovery, the low back muscle contraction should be carried out in a timely manner; 3 days after the operation, the ankle joint and knee joint rotation, back extension, and other exercises should be started; day 7 to 12 after the operation, the patients were instructed to exercise the hip and knee joint and the lower back muscles in a timely manner [8]. (4) Guidance on life rehabilitation: the patients should be instructed to maintain correct lying and sitting positions after surgery; in terms of diet, high-calcium, high-fiber, and high-protein foods should be abstained, and intake of calcium and vitamins should be added; (5) TCM syndrome differentiation believes lumbar discectomy and bone graft fusion and internal fixation patients are arthralgia disease (Qi stagnation and blood stasis type). Huoxue Shujin Recipe was used for supporting treatment: 15 g Sophora japonica, 15 g Tendon Radix, 25 g Pueraria Root, 10 g Myrrh, 15 g Stubbs, 5 g Turmeric, 15 g Angelica, 15 g Red Peony, 15 g Salvia, 15 g rhizoma chuanxiong, 15 g Corydalis Radix, 15 g Astragalus, and 5 g raw licorice. Totally, 7 doses were administered, 1 dose/d, splitting once in the morning and once in the evening with warm water. During this period, a stable and positive mood should be maintained to facilitate the recovery [9].

### 2.4. Observation Indicators

(1) Rehabilitation effect: markedly effective: the patient's activities returned to normal after nursing, and the clinical symptoms disappeared; effective: the patient's daily life basically resumed after nursing, and the clinical symptoms were greatly mitigated; ineffective: the patient's living ability did not improve after treatment, and the clinical symptoms did not mitigate or even aggravated. Total effective rate = (markedly effective + effective)/total number of cases × 100%. (2) Self-rating anxiety scale (SAS) and self-rating depression scale (SDS) scores: SAS and SDS were used to evaluate the psychological state of patients. 50–59 points were classified into mild anxiety, 60–69 points into moderate anxiety, and >70 points into severe anxiety. SDS score <53 was rated as no depression, 53–62 as mild depression, 63–72 as moderate depression, and >73 as severe depression. The lower the scores of the above indicators, the better the patient's psychological state. (3) Postoperative pain mitigation: the self-designed low back pain score scale of our hospital was used to detect the preoperative and postoperative pain of the patients. The full score of the scale was 100 points. The higher the score, the better the pain mitigation. (4) Nursing satisfaction: the “Nursing Satisfaction Questionnaire” designed by our hospital was used to score the patients. There are 20 questions in total, and the responses are summed to yield a total score ranged from 0–100 points <70 points are dissatisfied, 70–89 points are satisfied, and ≥90 points are very satisfied. Satisfaction = (very satisfied + satisfied)/total number of cases × 100%.

### 2.5. Statistical Analysis

Statistical analysis was performed using SPSS/ Statistics 18.0 software for Windows (SPSS Inc., Chicago, IL). The paired *t* test was performed to compare the differences in measurement data, while the chi-square test was performed to compare the differences in count data. All statistical significance levels were set at a *P* value of less than 0.05.

## 3. Results

### 3.1. Rehabilitation Effects

The postoperative rehabilitation effect of the rehabilitation group was significantly better than that of the routine group (*P* < 0.05), Table 1.

### 3.2. SAS and SDS Score

The fast rehabilitation nursing resulted in a notably lower postoperative SAS and SDS scores versus the routine nursing (*P* < 0.001), Table 2.

### 3.3. Postoperative Pain

The postoperative pain was significantly mitigated in the rehabilitation group when compared with the routine group (*P* < 0.001), Table 2.

### 3.4. Nursing Satisfaction

The fast rehabilitation nursing implemented in the rehabilitation group led to a remarkably higher nursing satisfaction of the patients (*P* < 0.001), Table 3.

## 4. Discussion

Lumbar intervertebral disc herniation is a common clinical disease in orthopaedics, and the contributors of this disease include heredity, congenital developmental abnormalities, external force injuries, and overwork [10]. The clinical manifestations of this disease are mainly weakened muscle strength, limitation of activities and low back pain, etc. [11, 12]. Although surgery is often used to treat lumbar intervertebral disc herniation with prominent efficacy [13], nursing service in clinical practice is imperative to greatly consolidate the treatment efficacy [14, 15]. Miyoshi et al. [16] have found that effective rehabilitation training for patients after surgery can not only significantly improve the effect of surgery, but also facilitate the prognosis of patients. Rapid rehabilitation nursing is an emerging nursing intervention model in recent years and is well-recognized by stimulating the patient's nerve functions to expand the nerve channel and guiding rehabilitation training to promote their blood circulation. As a result, it prevents the occurrence of nerve root adhesion in patients after surgery, thereby improving the prognosis of patients and the surgical efficacy [17].

In this study, we first compared the postoperative rehabilitation effect of the two groups of patients. The results showed that the postoperative rehabilitation effect of the patients in the rehabilitation group was significantly better than that of the patients in the routine group. Fast rehabilitation nursing for patients with lumbar intervertebral disc herniation can effectively improve the postoperative rehabilitation effect of patients. It is attributed to the fact that fast rehabilitation nursing will provide accurate and detailed rehabilitation guidance for patients after operation and help guide patients to carry out rehabilitation training; thereby, the rehabilitation effect can be improved [18], because most patients have insufficient understanding of their own diseases and fear of surgery-related trauma. Consequently, either the lack of knowledge or postoperative pain results in patients resistance to treatment, hugely hobbling the outcome of the surgery [19]. Notably, the combination of TCM medicines used in our study can nourish and relax tendons, nourish blood, and activate blood and treat both the symptoms and the essence, which can effectively mitigate the clinical symptoms of patients and greatly improve the quality of life of patients. Moreover, we compared the SAS score, SDS score, and back pain score of the two groups of patients and found that the postoperative SAS and SDS scores of the patients in the rehabilitation group were significantly lower than those in the routine group. These findings suggest that the fast recovery nursing could effectively relieve the patients' negative emotions and relieve the postoperative pain. The possible explanation may be that fast recovery nursing provides psychological support and psychological counseling to patients before surgery, creates a clean and tidy rehabilitation environment for patients after surgery, and relieves patients' body pain via other routes. [20]. Additionally, we compared the nursing satisfaction of the two groups of patients and found that the nursing mode in the rehabilitation group is associated with higher satisfaction, indicating that the fast rehabilitation nursing intervention has been extensively recognized by the patients and their families and further proving the practicability and reliability of rehabilitation nursing interventions [21].

## 5. Conclusion

Fast rehabilitation nursing mode intervention for lumbar disc herniation patients undergoing lumbar discectomy and bone graft fusion and internal fixation is a promising approach to improve the postoperative rehabilitation, mitigate postoperative pain, and minimize the occurrence of adverse reactions, with higher clinical nursing satisfaction. However, the number of patients included in this study was small, and a randomized multicenter study was not conducted. In the future, the number of patients included in the study will be expanded and the observation duration will be extended to obtain long-term clinical efficacy data to further verify the results.

## Figures and Tables

**Table 1:** Comparison of rehabilitation effects.

Groups	*n*	Markedly effective	Effective	Ineffective	Total (%)
Routine group	30	8	9	13	17 (56.7)
Rehabilitation group	30	21	8	1	29 (96.7)
*X* ^2^					12.468
*P*					＜0.05

**Table 2:** Comparison of SAS, SDS, and postoperative pain improvement (*x* ± *s*).

Groups	*n*	SAS		SDS		Back pain score	
		Before	After	Before	After	Before	After
Routine group	30	69.35 ± 2.36	58.63 ± 2.57	64.34 ± 3.21	55.62 ± 5.78	91.42 ± 5.31	42.59 ± 11.32
Rehabilitation group	30	69.41 ± 2.29	48.42 ± 2.67	64.40 ± 3.25	46.51 ± 5.49	91.55 ± 5.27	19.28 ± 12.65
*t*	—	0.115	17.425	0.083	7.228	0.11	8.685
*P*	—	0.909	＜0.001	0.934	＜0.001	0.913	＜0.001

**Table 3:** Comparison of nursing satisfaction.

Groups	*n*	Dissatisfied	Satisfied	Very satisfied	Total (%)
Routine group	30	14	8	8	16 (53.3)
Rehabilitation group	30	2	15	13	28 (93.3)
*X* ^2^	—	—	—	—	11.250
*P*	—	—	—	—	＜0.001

## Data Availability

No data were used to support this study.
